# The Addition of the Geriatric Nutritional Risk Index to the Prognostic Scoring Systems Did Not Improve Mortality Prediction in Trauma Patients in the Intensive Care Unit

**DOI:** 10.1155/2023/3768646

**Published:** 2023-05-31

**Authors:** Cheng-Shyuan Rau, Ching-Hua Tsai, Sheng-En Chou, Wei-Ti Su, Shiun-Yuan Hsu, Ching-Hua Hsieh

**Affiliations:** ^1^Department of Neurosurgery, Kaohsiung Chang Gung Memorial Hospital and Chang Gung University College of Medicine, Kaohsiung, Taiwan; ^2^Department of Trauma Surgery, Kaohsiung Chang Gung Memorial Hospital and Chang Gung University College of Medicine, Kaohsiung, Taiwan; ^3^Department of Plastic Surgery, Kaohsiung Chang Gung Memorial Hospital and Chang Gung University College of Medicine, Kaohsiung, Taiwan

## Abstract

**Background:**

Malnutrition is prevalent among critically ill patients and has been associated with a poor prognosis. This study sought to determine whether the addition of a nutritional indicator to the various variables of prognostic scoring models can improve the prediction of mortality among trauma patients in the intensive care unit (ICU).

**Methods:**

This study's cohort included 1,126 trauma patients hospitalized in the ICU between January 1, 2018, and December 31, 2021. Two nutritional indicators, the prognostic nutrition index (PNI), a calculation based on the serum albumin concentration and peripheral blood lymphocyte count, and the geriatric nutritional risk index (GNRI), a calculation based on the serum albumin concentration and the ratio of current body weight to ideal body weight, were examined for their association with the mortality outcome. The significant nutritional indicator was served as an additional variable in prognostic scoring models of the Trauma and Injury Severity Score (TRISS), the Acute Physiology and Chronic Health Evaluation (APACHE II), and the mortality prediction models (MPM II) at admission, 24, 48, and 72 h in the mortality outcome prediction. The predictive performance was determined by the area under the receiver operating characteristic curve.

**Results:**

Multivariate logistic regression revealed that GNRI (OR, 0.97; 95% CI, 0.96–0.99; *p*=0.007), but not PNI (OR, 0.99; 95% CI, 0.97–1.02; *p*=0.518), was independent risk factor for mortality. However, none of these predictive scoring models showed a significant improvement in prediction when the GNRI variable is incorporated.

**Conclusions:**

The addition of GNRI as a variable to the prognostic scoring models did not significantly enhance the performance of the predictors.

## 1. Background

Malnutrition is prevalent among severely injured patients, but it is frequently neglected [1]. The nutritional status of critically ill intensive care unit (ICU) patients may deteriorate rapidly after admission due to stress-induced catabolism, and the effects of malnutrition are likely to be exacerbated [2, 3]. Malnutrition is frequently associated with an increased risk of complications, a prolonged hospital stay, and a higher mortality rate in hospitalized patients [4, 5]. Additionally, malnourished patients would have a higher rate of ICU readmissions and infections [6].

Albumin levels, body mass index, muscular circumference, and questionnaires may determine nutritional status. However, there is no gold standard recommended for nutritional assessment [4]. Serum albumin level was affected by inflammatory processes, hydration, and hepatic or renal impairment [7]. The Subjective Global Assessment questionnaire classifies patients by medical history and physical examination [8] and is too complicated for quick filtering [9]. Mini Nutritional Assessment relies on the correctness of its questions and cannot be provided to elderly patients who have problems in communication, such as intubated ICU patients [10].

Some nutritional indicators which do not depend on a caregiver or patient's memory have been proposed to figure out a person's nutritional status. For example, the prognostic nutrition index (PNI) is calculated using the following formula: 10 serum albumin (g/dl) + 0.005 total lymphocyte count (/ul), in order to determine the nutritional status of surgical patients [11]. The PNI has been identified as an independent predictor of bad outcomes [12] and postoperative one-year mortality [13] after severe traumatic brain injury, and PNI increase was significantly associated with postoperative complications [14] in senior hip fracture patients [15, 16] and postoperative pulmonary complications in major burn patients [17]. Another nutritional indicator is the geriatric nutritional risk index (GNRI) [18], which is calculated as follows: [1.489 × albumin (g/dL) + 41.7 × (current body weight/ideal body weight)]. Hospitalized patients with GNRI have a strong correlation with handgrip strength, mid-upper arm muscle circumference, and arm muscle area [19]. GNRI has been effectively applied to a variety of illness, including heart failure [20], chronic obstructive pulmonary disease [21], chronic renal disease [22], and certain malignancy [23, 24] and also for the trauma patients [25–29].

It is essential to predict mortality in ICU trauma patients in order to enhance treatment planning and patient care. PNI and GNRI were both independent predictors of mortality in the hospital and after one year for ICU patients, according to a study [15]. However, given the fact that trauma patients exhibit a different picture of acute illness than those with chronic illness, the application of nutritional indicators to trauma patients must be validated beforehand. The Trauma and Injury Severity Score (TRISS) is the projection algorithm most commonly used to predict survival probability in trauma patients [16, 30, 31]. However, TRISS is not designed to predict mortality outcomes for ICU-admitted patients. Models of prognostic assessment have been developed specifically for ICU patients with critical illnesses. In our previous work, by forecasting the prognosis for 1,554 trauma patients in the ICU, we compared 11 prognostic scoring models and determined that the MPM II at 24 hours has the highest predictive efficacy [32]. This study aimed to determine whether the addition of a nutritional indicator to the variables of prognostic scoring models, such as TRISS, APACHE II, and MPM II, can result in a new model that more precisely predicts the mortality outcome of trauma patients in the ICU.

## 2. Methods

### 2.1. Ethical Statement

Before the study was conducted, Chang Gung Memorial Hospital's Institutional Review Board (IRB) authorized the procedure (approval numbers 202101617B0 and 202100201B0). Due to the retrospective nature of this investigation, the requirement that individual patients give their authorization to participate in the study was waived in accordance with the standards of the IRB.

### 2.2. Inclusion and Exclusion Criteria

Between January 1, 2018, and December 31, 2021, we obtained the enrolled data of 20,618 adult patients (aged 20 years) with all types of trauma from the hospital's Trauma Registry System [33]. (Figure 1). There were 3,061 patients admitted to the ICU. After excluding patients with burns (*n* = 63), hanging injuries (*n* = 5), drowning (*n* = 2), and those with incomplete laboratory data (*n* = 1,866), the study group consisted of 1,126 adult trauma patients with a critical illness.

### 2.3. Guidelines for Nutritional Support in the ICU

The ICU offered nutritional assistance to critically sick patients in accordance with the Society of Critical Care Medicine (SCCM) and American Society for Parenteral and Enteral Nutrition (ASPEN) recommendations [34, 35]. In summary, the guidelines recommend a daily energy intake of 25–30 kilocalories per kilogram of body weight, a daily protein intake of 1.2–2.0 grams per kilogram of body weight, enteral feeding whenever possible, regular nutritional status monitoring using a combination of clinical assessment and laboratory tests, and specialized nutrition support, including the use of immune-modulating nutrients and specialized formulas for patients.

### 2.4. Collection of the Medical Data

The hospital's trauma record was used to gather patients' medical information, including sex, age, prior comorbidities, Glasgow Coma Scale (GCS) score upon admission to the emergency department, Injury Severity Score (ISS), hospital stay in days, and in-hospital mortality. The preexisting comorbidities included diabetes mellitus (DM), hypertension (HTN), coronary artery disease (CAD), cerebrovascular accident (CVA), congested heart failure (CHF), and end-stage renal disease (ESRD). Laboratory data at the emergency room, including the count of white blood cells, lymphocytes, and platelets, levels of sodium, potassium, blood urine nitrogen, creatinine (Cr), bilirubin, hematocrit, oxygenation, arterial pH, and bicarbonate, were recorded. The albumin level measured in the emergency room or at the admission into ICU was recorded.

### 2.5. Calculation of the Scores

The PNI was computed using the following formula: 10 × serum albumin (g/dl) + 0.005 × total lymphocyte count (/ul). The GNRI was computed using the albumin amount and the ratio of body weight as per the following formula: [1.489 × albumin (g/dL) + 41.7 × (body weight/ideal body weight)]. The ideal body weight of men is (body height in cm-80) × 0.7, and that of women is (body height in cm-70) × 0.6. The TRISS primarily uses four variables—age; the Injury Severity Score (ISS); the Revised Trauma Score (RTS); and the injury mechanism. The ISS is an anatomical variable and RTS is a physiological variable value based on the patient's initial GCS score; systolic blood pressure; and respiratory rate. The injury mechanism defined by blunt or penetrating injuries to determine the probability of survival [36]. The TRISS was calculated based on a logarithmic regression equation: survival probability = 1/(1 + e − b), where *b* (penetrating injury) = −2.5355 + 0.9934 × RTS-0.0651 × ISS-1.1360 × age(index) and *b* (blunt injury) = −0.4499 + 0.8085 × RTS-0.0835 × ISS-1.7430 × age(index). In this formula, the age (index) is awarded 1 where patients above 55 and patients below 55 are awarded 0 [36]. The APACHE II and MPM II scores at admission were computed using factors collected at admission. According to the published algorithms, the MPM II score at 24 h, MPM II score at 48 h, and MPM II score at 72 h were calculated as proposed [37].

### 2.6. Statistical Analyses

For all statistical studies, Windows SPSS statistical software (version 23.0; IBM Inc., Chicago, IL, USA) was utilized. Categorical data were analyzed using Fisher's exact test or Pearson's 2 test, both of which are two-sided. Using the Kolmogorov–Smirnov test, the normalization of the continuously dispersed factors was assessed. Continuous data with a normal distribution were analyzed using analysis of variance with Bonferroni posthoc adjustment, whereas nonnormally distributed continuous data were analyzed using the Mann–Whitney *U* test. Continuous and discontinuous data are, respectively, represented as the mean standard deviation or median with interquartile range (IQR; Q1–Q3). Multivariate logistic regression analysis was utilized to find independent risk factors for death, with odds ratios (ORs) and 95% confidence intervals (CIs) being presented. Mortality within the institution was the main result of this research. With the inclusion of the nutritional status indicator along with the various variables of TRISS, APACHE II, and MPM II in a newly established regression model, the predictive performance was determined by the area under the receiver operating characteristic curve (AUCROC) utilizing the roc and roc.test function in the pROC package of *R* [38]. Because the TRISS measures the probability of survival, 1-TRISS was used to present the probability of mortality for a patient while plotting the receiver operating characteristic curves. A *p* value of less than 0.05 was regarded as statistically important. In all analyses, a two-tailed*p* value 0.05 was considered significant.

## 3. Results

### 3.1. Comparison between the Death and Survivor Group of Patients

The research population was divided into two categories, as shown in Table 1: death (*n* = 138) and survival (*n* = 988). There was no notable difference between the two categories in terms of gender predominance. Patients who died were considerably elderly and had a lower albumin concentration than those who survived. The level of lymphocytes did not vary significantly between the two groups. PNI and GNRI were markedly reduced in the mortality group compared to the survivor group (PNI: 41.6 ± 11.4 vs. 44.8 ± 9.4, *p* 0.001; GNRI: 94.4 ± 14.7 vs. 99.8 ± 12.5, *p* 0.001). Except for a considerably greater rate of CAD (15.2% vs. 8.7%, *p*=0.015), CHF (2.9% vs. 0.4%, *p*=0.001), and ESRD (8.7% vs. 2.9%, *p*=0.001) in the mortality group, there were no significant intergroup variations in the frequency of prior conditions. The mortality group had a significantly lower GCS score than the survival group (median (IQR): 7 [3–14, 17] vs. 15 [9–14, 17], *p* 0.001) but a significantly higher ISS score (median (IQR): 25 [15, 16, 22–33] vs. 20 [18–27], *p* 0.001). Patients in the mortality group had a lower inpatient length of stay (15.2 days vs. 23.5 days, *p* 0.001) than those in the survivor group.

### 3.2. Determinants of the Risk for Mortality

According to the findings presented in Table 2, multivariate logistic regression analysis of the imputed risk factors (age, PNI, GNRI, preexisting CAD, CHF, ESRD, and ISS) for mortality in univariate logistic regression analysis revealed that the age (OR, 1.02; 95% CI, 1.01–1.03; *p*=0.001), GNRI (OR, 0.97; 95% CI, 0.96–0.99; *p*=0.007), preexisting CHF (OR, 5.22; 95% CI, 1.14–23.96; *p*=0.033), ESRD (OR, 3.13; 95% CI, 1.43–6.81; *p*=0.004), and ISS (OR, 1.09; 95% CI, 1.07–1.11; *p* < 0.001) were significant independent risk factors for mortality. PNI was not the unique risk factor that was found to be contributing to the death of the patients.

### 3.3. Performance of the Prognostic Scoring Models with or without GNRI

Because GNRI, but not PNI, was a significant independent risk factor for patient death, a novel prediction method was developed by adding GNRI as a variable to the regression models of TRISS, APACHE II, and MPM II. Originally, the AUCs of these prognostic scoring models revealed that TRISS, APACHE II, MPM II at admission, MPM II at 24 h, MPM II at 48 h, and MPM II at 72 h had the AUC of 0.768, 0.823, 0.852, 0.871, 0.859, and 0841, respectively. The AUC of APACHE II, MPM II at admission, MPM II at 24 h, MPM II at 48 h, and MPM II at 72 h increased to 0.828, 0.859, 0.880, 0.868, and 0.851, respectively, when GNRI was included as a predictor in these prognostic scoring models. Although the AUC values in all models except TRISS showed a small increase, none of the models demonstrated a significant change when the GNRI variable was included (Figure 2).

## 4. Discussion

This study revealed that the nutritional indicator GNRI was a significant independent risk factor for mortality among ICU trauma patients. However, PNI was not identified as a significant risk factor that contributed to the patients' deaths. Moreover, when GNRI was included as a variable in these prognostic scoring models, none of the established models exhibited a significantly superior predictive performance than the original models.

The main reason that an addition of the nutritional indicator GNRI onto those prognostic scoring models did not significantly increase the prediction performance may be due to the characteristics of acute illness in these patients with a traumatic injury. The detrimental effect of malnutrition on the worse patient's outcome would be more prominent in the patients with chronic illness, considering that the mean hospital stay of those dead patients in this study is short and only 15.2 days. Given that the registered trauma database only records in-hospital mortality and not long-term mortality, it is possible that the long-term effect of nutritional status on a patient's mortality cannot be revealed. Moreover, in the acute condition, other factors, such as damage control, massive blood transfusion, resuscitation, and intervention surgery, may be more significant and paramount in determining the outcome of the patient.

The second reason may be attributed to that some variables used in these prognostic scoring models were, in part, associated with the nutritional status of the patients. The APACHE II uses age, mean arterial pressure, heart rate, respiratory rate, temperature, arterial blood pH, arterial oxygen pressure, serum sodium, serum potassium, serum creatinine, hematocrit, white blood cell count, and GCS to measure the severity of disease and predict death in critically ill patients [39–41]. The MPM II utilizes data on health status on admission, preexisting metastatic neoplasm or cirrhosis; acute diagnosis of infection, coma, and intracranial mass effect; physiological covariates of Cr levels, urine output, and partial pressure of oxygen; laboratory findings of prothrombin time; and additional factors such as mechanical ventilation and use of vasoactive drugs, to determine the outcome [42]. In APACHE II and MPM II, some input variables, including creatine, hemoglobin, and platelets, are correlated with the nutritional status of the patients. Creatinine levels, for instance, are influenced not only by age, exercise, stress, and renal disease but also by nutritional status [43–45]. In addition, the nutritional status would influence the hematological profile. A low hemoglobin level is associated with nutritional status, as caloric and protein restriction, iron, vitamin B12, and folic deficiency led to nutritional anemia [46, 47]. Patients with severe malnutrition also experience thrombocytopenia [48]. However, this theory did not explain why adding GNRI to TRISS, which had no nutritional status factor, did not improve prediction performance.

Third, all of the estimated models in this study were developed using logistic regression to predict patient death. Given the complexity of trauma etiology and biological expression in trauma patients, the limits of overfitting and multicollinearity of regression analysis may restrict the investigation of many complex explanatory factors. In this regard, machine learning may promise a promising future for dealing with complicated data and assisting in predictive diagnosis [49].

There are limitations to this research. Firstly, selection bias may have been present due to the retrospective nature of this research. Secondly, treatments such as surgery and resuscitation can produce a wide range of outcomes; however, when analyzing the data, we can only assume that these interventions produced consistent results. Thirdly, the recognized trauma database only documented patients who died while they were in the hospital; it did not document patients who were already dead when they arrived at the emergency department. As a result, there may be some selection bias when evaluating the results. In addition, the exclusion of patients who lacked certain test results at and during admission may have led to selection bias. Lastly, the group included in this research was confined to a singular trauma facility, restricting the generalizability of the results.

## 5. Conclusion

In ICU trauma patients, GNRI was an independent risk factor for death. However, adding GNRI to prognostic scoring models did not improve the predictive performance.

## Figures and Tables

**Figure 1:** Diagram illustrating the inclusion and exclusion criteria for adult trauma patients admitted to the intensive care unit.

**Figure 2:** The receiver operating characteristic curves and the area under the curve (AUC) of the prognostic scoring models with or without GNRI variable for trauma patients in the intensive care unit.

**Table 1:** Injury and patient characteristics of adult trauma patients who died and survived in the intensive care unit.

Variables	Death *n* = 138	Survival *n* = 988	OR (95% CI)	*p*
Sex				0.152
Male, *n* (%)	101 (73.2)	663 (67.1)	1.34 (0.90–2.00)	
Female, *n* (%)	37 (26.8)	325 (32.9)	0.75 (0.50–1.11)	
Age, years	62.0 ± 19.4	55.7 ± 19.1	—	<0.001
Albumin (g/dl)	3.1 ± 0.8	3.5 ± 0.7	—	<0.001
Lymphocyte (count)	2078.1 ± 1656.7	2007.4 ± 1468.8	—	0.602
PNI	41.6 ± 11.4	44.8 ± 9.4	—	<0.001
GNRI	94.4 ± 14.7	99.8 ± 12.5	—	<0.001
Comorbidities				
DM, *n* (%)	36 (26.1)	206 (20.9)	1.34 (0.89–2.02)	0.161
HTN, *n* (%)	57 (41.3)	329 (33.3)	1.41 (0.98–2.03)	0.063
CAD, *n* (%)	21 (15.2)	86 (8.7)	1.88 (1.13–3.15)	0.015
CHF, *n* (%)	4 (2.9)	4 (0.4)	7.34 (1.82–29.71)	0.001
CVA, *n* (%)	5 (3.6)	49 (5.0)	0.72 (0.28–1.84)	0.491
ESRD, *n* (%)	12 (8.7)	29 (2.9)	3.15 (1.57–6.33)	0.001
GCS, median (IQR)	7 (3–15)	15 (9–15)	—	<0.001
ISS, median (IQR)	25 (20–33)	20 (16–25)	—	<0.001
1–15	11 (8.0)	232 (23.5)	0.28 (0.15–0.53)	<0.001
16–24	33(23.9)	425 (43.0)	0.42 (0.28–0.63)	<0.001
≥25	94 (68.1)	331 (33.5)	4.24 (2.90–6.21)	<0.001
Hospital stay, days	15.2 ± 15.5	23.5 ± 18.1	—	<0.001

CAD = coronary artery disease; CHF = congestive heart failure; CI = confidence interval; CVA = cerebral vascular accident; DM = diabetes mellitus; ESRD = end-stage renal disease; GCS = Glasgow coma scale; GNRI = geriatric nutritional risk index; HTN = hypertension; IQR = interquartile range; ISS = injury severity score; OR = odds ratio; PNI = prognostic nutritional index.

**Table 2:** Univariate and multivariate analyses of the risk factors contributing to the mortality of trauma patients in the intensive care unit.

Variables	Univariate analysis		Multivariate analysis	
	OR (95% CI)	*p*	OR (95% CI)	*p*
Age, years	1.02 (1.01–1.03)	<0.001	1.02 (1.01–1.03)	0.001
PNI	0.96 (0.94–0.98)	<0.001	0.99 (0.97–1.02)	0.518
GNRI	0.97 (0.95–0.98)	<0.001	0.97 (0.96–0.99)	0.007
CAD, yes	1.88 (1.13–3.15)	0.016	1.57 (0.87–2.81)	0.131
CHF, yes	7.34 (1.82–29.71)	0.005	5.22 (1.14–23.96)	0.033
ESRD, yes	3.15 (1.57–6.33)	0.001	3.13 (1.43–6.81)	0.004
ISS	1.07 (1.06–1.09)	<0.001	1.09 (1.07–1.11)	<0.001

CAD = coronary artery disease; CHF = congestive heart failure; CI = confidence interval; ESRD = end-stage renal disease; GNRI = geriatric nutritional risk index; ISS = injury severity score; OR = odds ratio; PNI = prognostic nutritional index.

## Data Availability

The data supporting the current study are available from the corresponding author upon request.
